This article has been retracted.

# Study on the Changes of Liver and Kidney Function-Related Indicators and Clinical Significance in Patients with OSAHS

**DOI:** 10.1155/2022/9536617

**Published:** 2022-06-16

**Authors:** Rongyue Liu, Xiangdong Kong

**Affiliations:** ^1^Department of Otolaryngology, The First People's Hospital of Fuyang Hangzhou, Hangzhou 311400, Zhejiang, China; ^2^Department of Nephrology, The First People's Hospital of Fuyang Hangzhou, Hangzhou 311400, Zhejiang, China

## Abstract

**Purpose:**

To study the changes of liver and kidney function-related indexes in patients with obstructive sleep apnea hypopnea syndrome (OSAHS) and analyze their clinical significance.

**Method:**

Ninety OSAHS patients treated in our hospital from April 2019 to April 2021 were selected. According to the apnea-hypopnea Index (AHI), they were divided into mild OSAHS group (5 ≤ AHI < 15 times/h, 35 people), moderate OSAHS group (15 ≤ AHI < 30 times/h, 35 people), and severe OSAHS group (AHI ≥ 30 times/h, 20 people). In addition, 50 healthy people who underwent physical examination in our hospital at the same time were selected as the control group, and the liver and kidney function and polysomnography (PSG)-related indexes of the above subjects were detected, and the comparison between the groups was carried out.

**Result:**

The serum BUN and SCR levels of the severe group were significantly higher than those of the moderate group, the moderate group had significantly higher levels than the mild group, and the mild group had significantly higher levels than the control group (*P* < 0.05). The blood AST level of the severe group was significantly lower than that of the moderate group, the moderate group had a significantly lower level than the mild group, and the mild group had a significantly lower level than the control group (*P* < 0.05). The blood ALT level of the severe group was significantly higher than that of the moderate group, the moderate group had significantly a higher level than the mild group, and the mild group had a significantly higher level than the control group (*P* < 0.05). The proportions of abnormal liver and kidney function in the control group, mild group, moderate group, and severe group were significantly different (*P* < 0.05). The AHI of the severe group was significantly higher than that of the moderate group, the moderate group had a higher value than the mild group, and the mild group had a higher value than the control group (*P* < 0.05). The ASpO_2_ and MSpO_2_ of the severe group were significantly lower than those of the moderate group, the moderate group had significantly lower values than the mild group, and the mild group had significantly lower values than the control group (*P* < 0.05). Spearman correlation analysis showed that the liver and kidney function indexes of OSAHS patients were significantly correlated with PSG indexes (*P* < 0.05).

**Conclusion:**

Patients with OSAHS will have obvious liver and kidney dysfunction, and the monitoring of liver and kidney function in such patients should be strengthened. If abnormality occurs, early intervention is recommended.

## 1. Preface

Obstructive sleep apnea hypoventilation syndrome (OSAHS) is a sleep breathing disorder of unknown etiology [1], in which the main clinical manifestations include nocturnal snoring with apnea and daytime sleepiness. Clinical practice indicates that OSAHS is a potentially fatal sleep breathing disorder because of its tendency to cause recurrent episodes of nocturnal hypoxia and hypercapnia, which may lead to complications such as hypertension, coronary heart disease, diabetes mellitus, and cerebrovascular disease, and may even induce sudden death at night [2, 3]. Data from some large community-based population studies show that the prevalence of OSAS in recent years is about 4%–7.5% in men and 2% in women, and domestic epidemiological investigation suggests that the prevalence of OSAHS in adults is between 3% and 5% [4, 5].

In recent years, as research on OSAHS has intensified, more and more studies have pointed out that such patients may have concomitant hepatic and renal impairment [6]. Data show that about 51.7% of patients with OSAHS have concomitant polyuric symptoms, more than 30% of patients with OSAHS have concomitant chronic kidney disease, and some patients with OSAHS have decreased glomerular filtration rate [7]. A large number of studies have also concluded that although the site of OSAHS is the upper airway, the damage caused by the disorder is not limited to the upper airway itself. Systemic hypertension, atherosclerosis, coronary artery disease, arrhythmias, pulmonary hypertension, asthma, and Alzheimer's disease may be closely related to OSAHS [8]. Although the causal relationship between the above diseases and OSAHS is still being explored, an increasing number of scholars tend to define OSAHS as a multisystemic and multiorganic disease.

This study intends to investigate the changes of liver and kidney function-related indicators in patients with OSAHS by setting up a control group and attempts to investigate the necessity of liver and kidney function monitoring in patients with OSAHS, in order to provide clinical reference for improving the prognosis of patients with OSAHS.

## 2. Information and Method

### 2.1. General Information

Ninety patients with OSAHS treated in our hospital from April 2019 to April 2021 were selected. They were divided into mild OSAHS group (5 ≤ AHI < 15 times/h, 35 patients), moderate OSAHS group (15 ≤ AHI < 30 times/h, 35 patients), and severe OSAHS group (AHI ≥ 30 times/h, 20 patients) according to apnea-hypopnea index (AHI). 50 healthy individuals who underwent physical examination in our hospital at the same time were selected as the control group.

#### 2.1.1. Inclusion Criteria

(1) Patients with OSAHS met clinical diagnostic criteria [9] and presented with appropriate clinical symptoms. (2) Patients were conscious and able to cooperate with the study. (3) Case data were complete and available. (4) Patients have good compliance with the study. (5) Patients have signed informed consent. (6) AHI score ≥ 5. (7) The study was approved by the ethics association to be conducted.

#### 2.1.2. Exclusion Criteria

(1) Patients have combined psychiatric disorders. (2) Patients have combined malignant neoplasm. (3) Patients have combined liver and kidney dysfunction. (4) Patients have combined autoimmune diseases. (5) Patients have combined pulmonary diseases. (6) Patients have complicated blood system diseases, hyperthyroidism, hypothyroidism, etc. (7) Patients have been taking drugs with impaired liver and kidney function within the last 1 month.

### 2.2. Intervention Method

(1) Sleep monitoring: all patients in the study group completed PSG monitoring, and no sleeping pills or alcohol, tea, coffee, etc. could be taken within 24 h before the test. The subjects were mainly monitored for sleep structure, breathing, snoring, and body position, and their sleep conditions were judged according to the American Academy of Sleep Medicine sleep and its related events (AASM) criteria [10], and their AHI, ASpO_2_, and MSpO_2_ indicators were recorded. (2) Fasting elbow venous blood samples were collected from all subjects, and liver and kidney functions were tested by automatic biochemical analyzers, including AST and ALT for liver functions and BUN and SCr for kidney functions.

### 2.3. Observation Indicators and Evaluation Criteria

The patients in the study group were distinguished into mild OSAHS group (5 ≤ AHI < 15 times/h, 35 cases), moderate OSAHS group (15 ≤ AHI < 30 times/h, 35 cases), and severe OSAHS group (AHI ≥ 30 times/h, 20 cases), according to the AHI index [11]. The differences in liver and kidney function and PSG-related indicators between the above three groups and control individuals were compared between groups, and the correlation between liver and kidney function indicators of patients with OSAHS and their PSG indicators was also analyzed.

### 2.4. Statistical Method

Spss22.0 statistical software was selected to analyze the data collected in the study, in which the measured data were expressed as (standard deviation of mean value ± for standard deviation) normal distribution and chi square test, t-test was used for the differences between data groups that conform to normal distribution or chi square distribution, and Mann Whitney u test was used for statistics of data with inconsistent variance. The difference between groups was tested using the chi-square test, and the difference was considered statistically significant at *P* < 0.05. The GraphPad Prism 8.3 was used in this study [12].

## 3. Result

### 3.1. Comparison of Baseline Information between Groups of Patients

Age, gender, BMI, blood pressure, blood test-related indicators, and respiratory sleep monitoring-related indicators were included in the study and carried out to compare the difference between groups, and the result showed that the difference between groups in age, gender, BMI, blood pressure, blood glucose, total cholesterol, and triglycerides in several groups were not statistically significant (*P* < 0.05), suggesting that the groups were better comparable (see Table 1).

### 3.2. Comparison of Renal Function Indicators between Groups of Patients

The results showed that the serum BUN and SCr levels of patients in the severe group were significantly higher than those in the moderate group, the moderate group had significantly higher levels than the mild group, and the mild group had significantly higher levels than the control group, and the differences between the groups were statistically significant (*P* < 0.05) (see Table 2 and Figure 1).

The serum BUN and SCr levels of patients in the severe group were significantly higher than those in the moderate group, the moderate group had significantly higher levels than the mild group, and the mild group had significantly higher levels than the control group, and the differences of the above indicators were statistically significant when comparing between groups (*P* < 0.05). # represents a statistically significant difference between groups comparing the same index.

### 3.3. Comparison of Liver Function Indicators between Groups of Patients

The AST and ALT level of blood samples from patients in the mild group, moderate group, severe group, and control group were tested and compared between the groups. The ALT level of blood samples of patients in the severe group was significantly higher than that in the moderate group, the moderate group had a significantly higher level than the mild group, and the mild group had a significantly higher level than the control group. The difference of the above indicators were statistically significant when comparing between groups (*P* < 0.05) (see Table 3 and Figure 2).

The AST level of blood samples of patients in the severe group were significantly lower than those in the moderate group, the moderate group had significantly a lower level than the mild group, and the mild group had a significantly lower level than the control group. The difference of above indicators were statistically significant when comparing between groups (*P* < 0.05). The ALT level of blood samples of patients in the severe group was significantly higher than that in the moderate group, the moderate group had a significantly higher level than the mild group, and the mild group had a significantly higher level than the control group. The difference of above indicators were statistically significant when comparing between groups (*P* < 0.05). # represents a statistically significant difference between groups comparing the same index.

### 3.4. Comparison of the Rate of Abnormal Liver and Kidney Function in Each Group of Patients

The percentage of liver and kidney function abnormalities in each group was compared between groups, and the results showed that there were large differences in the ratio of liver and kidney function abnormalities in the control, mild, moderate, and severe groups. The comparison between groups showed that the percentage of liver and kidney function abnormalities in the moderate and severe groups was significantly higher than that in the mild and control groups, and the difference in some indicators were statistically significant (*P* < 0.05) (see Table 4).

### 3.5. Comparison of PSG-Related Indicators between Groups of Patients

The PSG test was performed on each group of patients separately, and the indices of AHI, ASpO_2_, and MSpO_2_ of the subjects were tested and compared between the groups. The ASpO_2_ and MSpO_2_ of patients in the severe group were significantly lower than those in the moderate group, the moderate group had significantly lower values than the mild group, and the mild group had significantly lower values than the control group. The difference between the groups were statistically significant (*P* < 0.05) (see Table 5 and Figure 3).

Comparison showed that the AHI of patients in the severe group was significantly higher than that in the moderate group, the moderate group had a higher value than the mild group, and the mild group had a higher value than the control group. The difference between the groups was statistically significant (*P* < 0.05). The ASpO_2_ and MSpO_2_ of patients in the severe group were significantly lower than those in the moderate group, the moderate group had significantly lower values than the mild group, and the mild group had significantly lower values than the control group. The difference between the groups were statistically significant (*P* < 0.05). # represents a statistically significant difference between groups comparing the same index.

### 3.6. Correlation Analysis of Liver and Kidney Function Indicators with PSG Indicators in Patients with OSAHS

Spearman analysis was performed on the correlation between liver function indicators (AST and ALT), kidney function indicators (BUN and SCr) and PSG indicators (AHI, ASpO_2_, and MSpO_2_) in patients with OSAHS. The results showed that AST showed significant correlation with AHI, ASpO_2_, and MSpO_2_ (*r* = −0.726, 0.556, 0.519, *P* < 0.05), ALT showed significant correlation with AHI, ASpO_2_, and MSpO_2_ (*r* = 0.712, −0.772, −0.549, *P* < 0.05), and BUN showed significant correlations with AHI, ASpO_2,_ and MSpO_2_ (*r* = 0.459, −0.771, −0.627, *P* < 0.05), and SCr showed significant correlations with AHI, ASpO_2,_ and MSpO_2_ (*r* = 0.819, −0.728, −0.711, *P* < 0.05) (see Table 6).

## 4. Discussion

Since the 1970s, there has been increasing concern about OSAHS worldwide [13]. Overseas epidemiological surveys for snoring and OSAHS began 20 years ago in the form of questionnaires and telephone calls, and some of these patients were even monitored for sleep breathing throughout the night. It was concluded that the prevalence of OSAHS in individuals under 65 years was about 0.3%–1%, with men prevalence significantly higher than that of women [14]. Less epidemiological investigation has been conducted for OSAS in China, but the prevalence of the disorder has shown a significant increase in recent years with the rise in life and work stress among the population [15].

Medical practitioners believe that patients with OSAHS are superior to the collapse of the upper airway during sleep, prone to apnea and hypoventilation, followed by a series of changes such as endothelial damage, sleep structural fragmentation, endocrine hormone abnormalities, and inflammatory reactions, which can cause safety threats to the circulatory, neurological, metabolic, endocrine, respiratory, urinary, hematological, and other systemic systems of patients, especially cardiovascular, hepatic, and renal function damage are the most [16, 17]. Studies have confirmed the independent correlation between OSAS and cardiovascular diseases, and patients with OSAHS are significantly more likely to develop hypertension, stroke, pulmonary hypertension, chronic kidney disease, and other disorders [18, 19].

In this study, we investigated the changes in liver and kidney function in patients with OSAHS by setting up a control group, and the results showed that compared with the control group, patients with OSAHS showed a significant decrease in AST, a significant increase in ALT, and a significant increase in BUN and SCr. Both indicators of kidney function and the changes were also closely related to the condition of OSAHS.

In a study of 230 patients with OSAHS [20], the level of reactive oxygen species, hypoxia-inducible factor-1*α*, nitric oxide, urea nitrogen, creatinine, and uric acid in the serum of patients with moderate to severe OSAHS were significantly different from those of patients with mild OSAHS and normal controls, which is believed to be due to the presence of chronic hypoxia in patients with OSAHS. Chronic hypoxia, which in turn induces renal impairment, can be considered as a potential risk factor for chronic renal insufficiency in OSAHS. In a study conducted on 50 patients with OSAHS and 40 healthy controls [21], it was found that the level of ALT, TC, AST, BUN, and SCr were abnormally elevated in patients with mild to moderate and severe OSAHS compared to normal controls, while the elevation of AST and SCr was particularly severe in patients with severe OSAHS. In this study, we analyzed that AST and ALT can reflect the integrity of hepatocyte membrane or mitochondria, and their serum concentrations can reflect the damage status of hepatocytes more sensitively; thus, they are often used in clinical screening for impaired liver function [22]. BUN and SCr are both common indicators of renal function examination in clinical practice, among which SCr can also reflect glomerular filtration rate [23]. Due to impaired airway function and long-term hypoxia, several studies have confirmed that OSAHS is an independent risk factor for diseases such as cardiac arrhythmia, congestive heart failure, insulin resistance, and hyperlipidemia, and also a risk factor for the development of chronic kidney injury.

Continued exacerbation of OSAHS without better control will induce and aggravate the decline of liver and kidney function and eventually lead to the development of liver and kidney impairment [24]. Patients with OSAHS can develop significant liver and kidney dysfunction, and monitoring of liver and kidney function in such patients should be strengthened, and early implementation of interventional therapy is recommended in case of abnormalities. The limitations of this study are as follows: (1) There were more men than women in the study, and gender bias may have had an impact on the results. (2) Changes in the abovementioned indicators in patients with OSAHS after the intervention were not studied. (3) Detailed mechanisms of liver and kidney function impairment in OSAHS patients were not analyzed. Revisions and improvements are planned for later stages. In this paper, the authors analyzed that, in addition to the above mechanisms, there may be another reason for OSAHS-induced liver and kidney injury, namely, OSAHS causes the body to be in a state of inflammatory imbalance. Many studies have pointed out that the levels of superoxide dismutase, interleukin-2, and tumor necrosis factor are significantly elevated in patients with severe OSAHS, analyzing that OSAHS leads to a disturbance in the immune imbalance of the organism [25], and the present study suggests that this may also be related to the development of OSAHS, and further in-depth study of the mechanism is needed.

## Figures and Tables

**Figure 1:** Comparison of renal function indicators among groups.

**Figure 2:** Comparison of liver function indicators of patients in each group.

**Figure 3:** Comparison of PSG-related indicators among groups of patients.

**Table 1:** Comparison of baseline information of patients in different groups ($\bar{x}\pm s$)/(*n* (%)).

General clinical information		Mild group (*n* = 35)	Moderate group (*n* = 35)	Severe group (*n* = 20)	Control group (*n* = 50)	*F*	*P* value
Gender	Male	20	19	8	25	1.211	0.723
	Female	15	16	12	25		
Average age (years)		49.89 ± 3.22	50.19 ± 2.98	50.11 ± 2.38	49.78 ± 3.89	0.123	0.946
Average BMI (kg/m^2^)		23.29 ± 2.39	23.41 ± 2.09	23.89 ± 2.11	23.78 ± 2.01	0.571	0.635
Systolic blood pressure (mmHg)		124.38 ± 10.19	123.98 ± 9.98	123.78 ± 10.31	124.08 ± 10.78	0.016	0.997
Diastolic blood pressure (mmHg)		78.98 ± 5.44	79.01 ± 4.98	79.13 ± 5.01	79.33 ± 4.87	0.043	0.988
Blood glucose (mmol/L)		4.98 ± 0.98	5.01 ± 0.89	5.04 ± 0.87	4.99 ± 1.01	0.020	0.996
Total cholesterol (mmol/L)		4.49 ± 0.43	4.53 ± 0.39	4.51 ± 0.33	4.59 ± 0.29	0.6	0.616
Triglycerides (mmol/L)		2.29 ± 0.32	2.30 ± 0.29	2.34 ± 0.31	2.33 ± 0.28	0.201	0.896
High-density lipoprotein (mmol/L)		1.12 ± 0.12	1.14 ± 0.09	1.15 ± 0.12	1.18 ± 0.14	1.813	0.148
Low-density lipoprotein (mmol/L)		2.87 ± 0.54	2.78 ± 0.49	2.91 ± 0.31	2.84 ± 0.21	0.523	0.667

**Table 2:** Comparison of renal function indicators among patients in each group ($\bar{x}\pm s$).

Group	Number of cases	BUN (mmol/L)	SCr (*μ*mol/L)
Mild group	35	5.11 ± 0.45^①②③^	83.22 ± 4.22^①②③^
Moderate group	35	5.39 ± 0.39^①②^	88.98 ± 3.98^①②^
Severe group	20	5.78 ± 0.29^①^	93.29 ± 4.01^①^
Control group	50	4.68 ± 0.33	76.11 ± 3.98
*F*	—	50.003	116.111
*P* value	—	<0.001	<0.001

Compared with the control group, ^①^*P* < 0.05; compared with the severe group, ^②^*P* < 0.05; compared with the moderate group, ^③^*P* < 0.05.

**Table 3:** Comparison of liver function indicators among patients in each group ($\bar{x}\pm s$).

Group	Number of cases	AST (U/L)	ALT (U/L)
Mild group	35	21.27 ± 3.22 ^①②③^	33.18 ± 3.20^①②③^
Moderate group	35	25.03 ± 2.39^①②^	40.11 ± 4.10^①②^
Severe group	20	27.19 ± 3.01^①^	46.18 ± 3.98^①^
Control group	50	29.89 ± 4.33	22.91 ± 3.20
*F*	—	367.330	271.976
*P* value	—	<0.001	<0.001

Compared with the control group, ^①^*P* < 0.05; compared with the severe group, ^②^*P* < 0.05; compared with the moderate group, ^③^*P* < 0.05.

**Table 4:** Comparison of abnormal liver and kidney function rates among groups (*n* (%)).

Observed indicators		Mild group (*n* = 35)	Moderate group (*n* = 35)	Severe group (*n* = 20)	Control group (*n* = 50)
Liver function	AST	0 (0.00)	4 (11.43)^①②^	5 (20.00)^①②^	0 (0.00)
	ALT	3 (8.57)	8 (22.86)^①^	10 (50.00)^①②^	1 (2.00)

Renal function	BUN	4 (11.43)	7 (20.00)^①^	8 (40.00)^①^	1 (2.00)
	SCr	2 (5.71)	6 (17.14)^①^	9 (45.00)^①②^	1 (2.00)

Compared with the control group, ^①^*P* < 0.05; compared with the mild group, ^②^*P* < 0.05.

**Table 5:** Comparison of PSG-related indicators among patients in each group ($\bar{x}\pm s$).

Group	Number of cases	AHI (times/h)	ASpO_2_ (%)	MSpO_2_ (%)
Mild group	35	13.22 ± 1.98^①②③^	96.18 ± 3.49^①②③^	83.18 ± 5.01^①②③^
Moderate group	35	23.89 ± 3.21^①②^	93.29 ± 4.01^①②^	76.18 ± 4.22^①②^
Severe group	20	60.19 ± 5.41^①^	90.19 ± 2.30^①^	64.29 ± 4.30^①^
Control group	50	3.98 ± 0.43	99.28 ± 3.90	89.18 ± 3.49
*F*	—	240.465	36.619	189.593
*P* value	—	<0.001	<0.001	<0.001

Compared with the control group, ^①^*P* < 0.05; compared with the severe group, ^②^*P* < 0.05; compared with the moderate group, ^③^*P* < 0.05.

**Table 6:** Correlation analysis of liver and kidney function indicators with PSG indicators in patients with OSAHS.

Indicators	AST	ALT	BUN	SCr	AHI	ASpO_2_	MSpO_2_
AST	—	—	—	—	−0.726	0.556	0.519
ALT	—	—	—	—	0.712	−0.772	−0.549
BUN	—	—	—	—	0.459	−0.771	−0.627
SCr	—	—	—	—	0.819	−0.728	−0.711
AHI	−0.726	0.712	0.459	0.819	—	—	—
ASpO_2_	0.556	−0.772	−0.771	−0.728	—	—	—
MSpO_2_	0.519	−0.549	−0.627	−0.711	—		—

## Data Availability

The raw data supporting the conclusions of this article will be made available by the authors, without undue reservation.
